# A Critical HA1 Neutralizing Domain of H5N1 Influenza in an Optimal Conformation Induces Strong Cross-Protection

**DOI:** 10.1371/journal.pone.0053568

**Published:** 2013-01-08

**Authors:** Lanying Du, Guangyu Zhao, Shihui Sun, Xiujuan Zhang, Xiaojun Zhou, Yan Guo, Ye Li, Yusen Zhou, Shibo Jiang

**Affiliations:** 1 Lindsley F. Kimball Research Institute, New York Blood Center, New York, New York, United States of America; 2 State Key Laboratory of Pathogen and Biosecurity, Beijing Institute of Microbiology and Epidemiology, Beijing, China; 3 School of Medical Laboratory Science, Wenzhou Medical College, Wenzhou, Zhejiang, China; 4 Key Laboratory of Medical Molecular Virology of Ministries of Education and Health, Shanghai Medical College and Institute of Medical Microbiology, Fudan University, Shanghai, China; Fudan University, China

## Abstract

The highly pathogenic avian influenza (HPAI) H5N1 viruses, especially the laboratory-generated H5N1 mutants, have demonstrated the potential to cross the species barrier and infect mammals and humans. Consequently, the design of an effective and safe anti-H5N1 vaccine is essential. We previously demonstrated that the full-length hemagglutinin 1 (HA1) could induce significant neutralizing antibody response and protection. Here, we intended to identify the critical neutralizing domain (CND) in an optimal conformation that can elicit strong cross-neutralizing antibodies and protection against divergent H5N1 strains. We thus constructed six recombinant proteins covering different regions of HA1 of A/Anhui/1/2005(H5N1), each of which was fused with foldon (Fd) and Fc of human IgG. We found that the critical fragment fused with Fd/Fc (HA-13–263-Fdc, H5 numbering) that could elicit the strongest neutralizing antibody response is located in the N-terminal region of HA1 (residues 13–263), which covers the receptor-binding domain (RBD, residues 112–263). We then constructed three additional recombinants fused with Fd plus His tag (HA-13–263-Fd-His), Fc only (HA-13–263-Fc), and His tag only (HA-13–263-His), respectively. We found that the HA-13–263-Fdc, which formed an oligomeric conformation, induced the strongest neutralizing antibody response and cross-protection against challenges of two tested H5N1 virus strains covering clade 1: A/VietNam/1194/2004 (VN/1194) or clade 2.3.4: A/Shenzhen/406H/06 (SZ/406H), while HA-13–263-Fc dimer and HA-13–263-Fd-His trimer elicited higher neutralizing antibody response and protection than HA-13–263-His monomer. These results suggest that the oligomeric form of the CND containing the RBD can be further developed as an effective and safe vaccine for cross-protection against divergent strains of H5N1 viruses.

## Introduction

The highly pathogenic avian influenza (HPAI) A/H5N1 is considered a significant threat for the next influenza pandemic. The genetic variability of this virus makes it an unprecedented risk for the global spread of the new virus strains. Although human-to-human transmission of this virus has been very rare, this phenomenon is challenged by recent successful transmission of the laboratory-generated mutant H5N1 virus [1], [2]. Either insertion of mutated hemagglutinin (HA) gene of H5N1 into a 2009 pandemic H1N1 strain or selection of a H5N1 virus strain with five mutations results in the generation of viruses able to confer efficient transmissibility among ferrets, an animal model closely resembling humans in flu studies [1], [2]. Since the H5N1 virus has shown case fatality rate around 60% with 359 deaths among a total 608 human infections reported to WHO as of August 10, 2012 (http://www.who.int/influenza/human_animal_interface/EN_GIP_20120810CumulativeNumberH5N1cases.pdf), suitable measures and novel strategies are urgently needed to prevent the potential threat caused by H5N1 viruses with divergent strains. Effective vaccines would play a key role in preventing the dire predictions noted above.

Among all influenza virus proteins, HA, a major antigen on the viral surface, serves as an important protein in inducing neutralizing antibodies and cross-protection [3]. The HA-specific antibodies could neutralize infectivity of the HPAI N5N1 viruses by interacting with the receptor binding domain (RBD) or blocking conformational rearrangement associated with membrane fusion [4], [5]. It has been reported that antibodies to virus HA protein mediate heterosubtype neutralizing responses to A/H5N1 viruses in healthy volunteers exposed to H5N1 [6]. Animals vaccinated with HA DNA also show higher neutralizing antibody responses and/or better protection than NA, NP, or M2 DNA vaccines against challenges with homologous or heterologous H5N1 viruses [7]. A tri-clade DNA vaccine encoding HA of clade 0, 2.3.2.1 and 7.2 elicits broadly neutralizing antibody responses against H5 clades and subclades and protects mice against heterologous H5N1 challenge [8]. Therefore, based on its strong ability to induce neutralizing antibodies and protection, HA is considered a primary target for designing effective vaccines against H5N1 virus infection.

The HA protein is a homotrimer. Each of its single-chain monomers initially synthesizes as a precursor polypeptide, HA0, which is then cleaved by host proteases into two subunits, HA1 and HA2 [9]. The RBD of H5N1 viruses is located at the N-terminal HA1 region, covering amino acid residues from around 112 to 263 [10]–[12]. A reassortant virus, comprising four mutations (N158D/N224K/Q226L/T318I) of H5 HA (three of which are in RBD) and seven gene segments from a 2009 pandemic H1N1 virus, may preferentially recognize human-type receptors and transmit efficiently in ferrets, emphasizing the importance of HA, particularly RBD, in receptor binding specificity, virus infection and transmission. The success of laboratory-generated transmissible mutant virus and continual evolvement of H5N1 viruses in the nature significantly increase the possibility for emerging receptor-binding variants of H5N1 viruses with pandemic potential [1]. Therefore, identification of the critical neutralizing domain (CND) of HA, particularly RBD, will be of great importance to develop efficacious and safe vaccines against variant H5N1 virus.

It should be noted that the vaccines designed to maintain suitable conformational structure of HA are expected to produce stronger immune responses. In fact, it has been revealed that 1) the trimeric form of HA may significantly improve immunogenicity over that of monomeric HA in vaccinated mice against influenza A virus (IAV) infection, and 2) a H5N1 virus-like particle vaccine elicits cross-reactive neutralizing antibodies preferentially binding to the oligomeric form of influenza virus HA in humans [13], [14].

Previously, we have shown that a recombinant vaccine covering the full-length HA1 region of H5N1 induced neutralizing activity against divergent strains of H5N1 influenza virus [15], suggesting that the HA1 subunit of HA protein plays significant roles against virus infection and serves as an attractive target for vaccine development. However, to design an effective and safe HA1-based vaccine, it is essential to identify the critical neutralizing domain in HA1, especially in the RBD of H5N1 HA protein. For example, we have designed a highly effective and safe vaccine against severe acute respiratory syndrome (SARS) coronavirus (SARS-CoV) using the critical neutralizing domain in the RBD of the viral spike (S) protein, a class I fusion glycoprotein similar to the HA of influenza virus, and shown its efficacy against SARS virus infections [16]–[19]. We therefore carried out an initial study by constructing a series of truncated fragments covering different lengths of the HA1 of H5N1 virus, including the full-length or partial-length RBD or no RBD, and containing foldon (Fd) trimeric motif and Fc of human IgG at the C-termini in order to identify the CND of HA1 that can induce neutralizing antibodies. We then used the identified CND with or without Fd or Fc to construct a series of new recombinants with different conformations, for the purpose of identifying an appropriate conformation of the CND in HA1 that can induce the strongest protective immunity against divergent strains of H5N1 virus.

## Results

### Expression and Characterization of Truncated HA1 Protein Fragments

In this study, we constructed six recombinant proteins covering different lengths of HA1 of H5N1 virus, including full-length RBD (HA-112–263, HA-38–263, and HA-13–263), or partial-length RBD (HA-13–158 and HA-13–218) or no RBD (HA-13–90), and containing Fd and Fc at the C-termini (Fig. 1). All six constructs were able to express soluble proteins in the culture supernatant of transfected 293T cells, maintaining high expression with strong purity, as shown in SDS-PAGE (Fig. 2A). The expressed proteins were shown as monomers in the boiled sample lines, but the molecular weight shown in the non-boiled proteins is around 2-fold higher than that of the boiled samples after addition of the sample buffer containing 2% SDS and 1% 2-mercaptoethanol reducing agent and migration of the gels in the presence of 0.1% SDS, indicating that all expressed proteins fused with Fd and Fc formed suitable conformational structures similar to dimers in the reducing SDS-PAGE (Fig. 2A). In addition, Western blot results revealed strong bands corresponding to the relative molecular weight of the recombinant proteins, demonstrating that all proteins were recognized by a HA1-specific mAb (Fig. 2B).

**Figure 1:** Construction of recombinant truncated HA1 protein fragments fused with Fd and Fc. (A) Schematic structure of HA protein of A/Anhui/1/2005 (H5N1 HA). SP, signal peptide. FP, fusion peptide. HA1-Fdc protein was previously expressed covering HA residues +3–322 [15], corresponding to residues 13–325 of H5 numbering as described in the published literature [9], [20], [21]. (B) Truncated HA fragments covering various lengths of HA1 were constructed by fusing HA1 fragments with Fd and Fc. Each fragment contains IL2ss signal peptide at the 5′ terminus for the purpose of leading expressed proteins to the culture supernatant. The predicted RBD region was indicated in black.

**Figure 2:** SDS-PAGE and Western blot analysis of expressed proteins containing truncated HA1 fragments. Protein samples were either boiled at 95°C for 5 min, or not boiled, followed by addition of 6× SDS-PAGE sample buffer. SDS-PAGE with Coomassie Blue staining was then run (A), as well as Western blot (B) by using a HA1-specific mAb. The protein molecular weight marker (kDa) (Invitrogen) is indicated on the left.

### Fragment Containing Residues 13–263 of HA1 Induced the Strongest Neutralizing Antibody Responses Compared with other Truncated HA1 Proteins

All six truncated protein fragments were used to immunize mice, as described in Materials and Methods, and sera were collected 10 days post-last vaccination to detect HA1-specific antibody responses and neutralizing activity against homologous H5N1 virus. As shown in Fig. 3A, all protein fragments induced high HA1-specific IgG antibodies in the vaccinated mice, with no significant differences being detected in the sera collected from any vaccinated group. An average endpoint antibody titer of 1 : 2.1 × 10^8^ was detected in the sera of mice vaccinated with all six proteins (Fig. 3B), suggesting that these truncated HA1 protein fragments containing suitable conformation have high immunogenicity in eliciting potent antibody responses in the vaccinated mice.

**Figure 3:** Detection of antibody responses and evaluation of neutralizing activity for sera of mice vaccinated with truncated HA1. Sera from 10 days post-last vaccination were used for the detection. (A) Detection of sera IgG antibody responses by ELISA respectively coated with truncated HA1 protein fragments with the serum dilution at 1∶12800. The data are presented as mean A450± standard deviation (SD) of five mice per group. (B) ELISA detection of IgG binding ability to the truncated HA1 protein fragments. The data are presented as mean A450± SD of five mice per group at various dilution points. (C) Neutralizing antibody titers against HA of homologous strain A/Anhui/1/2005(H5N1) (AH-HA, clade 2.3.4) of H5N1 pseudovirus. The data are presented as mean 50% neutralizing antibody titer (NT_50_) ± SD from five mice per group. * indicates significant difference (*P*<0.05) between HA-13–263-Fdc vaccination group and other groups.

The neutralizing activity induced by these protein fragments was further evaluated in the collected mouse sera against homologous AH-HA strain of H5N1 pseudovirus. As indicated in Fig. 3C, the HA-13–263-Fdc vaccinated group elicited very strong neutralizing antibody response against AH-HA H5N1 pseudovirus, reaching a titer of 1∶8.6 × 10^4^±5.7 × 10^4^, which is significantly higher (*P<*0.05) than that induced by the groups vaccinated with the other five truncated protein fragments, including residues 112–263, 38–263, 13–90, 13–158, and 13–218 of HA1 region. These results suggest that the protein fragment containing residues 13–263 of HA1 is the CND in HA1 that could induce the strongest neutralizing antibody response and its fusion protein containing Fd and Fc (HA-13–263-Fdc) may be an ideal immunogen for inducing highly potent neutralizing responses against H5N1 virus infection.

### Fragment Containing Residues 13–263 of HA1 Fused with Fd and/or Fc Tags was able to form Polymeric Conformational Structures

Based on the identified HA-13–263 neutralizing region, we constructed three additional recombinants, respectively fused with Fc (HA-13–263-Fc), Fd-His (HA-13–263-Fd-His), or His (HA-13–263-His) (Fig. 4A), and expressed these proteins in the culture supernatant of 293T cells, followed by characterizing the ability of this neutralizing HA fragment to form different conformational structures of HA. As shown in SDS-PAGE (Fig. 4B), one clear band was observed in the non-boiled samples of HA-13–263-Fdc and HA-13–263-Fc with a molecular weight higher (almost 2-fold) than observed in the boiled samples (monomers), suggesting that HA-13–263 mainly form dimeric conformational structures. In addition, the top band from the non-boiled HA-13–263-Fd-His sample line had a molecular weight almost 3-fold greater than the boiled line (monomer), revealing that HA-13–263 fused with Fd mainly form trimeric conformational structure. In the line of HA-13–263-His protein, similar bands with almost identical molecular weight were detected in both boiled and non-boiled conditions, indicating that HA-13–263 fragment alone maintained a monomeric form. Accordingly, these particular bands shown in SDS-PAGE were further confirmed in Western blot analysis by a HA1-specific mAb developed in our laboratory (Fig. 4C).

**Figure 4:** Construction of protein fragments containing HA-13–263 with or without Fd or Fc and analysis of protein expression. (A) Proteins containing residues of HA-13–263 with Fc (HA-13–263-Fc), with Fd (HA-13–263-Fd-His), or without fusion with Fd and Fc (HA-13–263-His) were constructed. Purified proteins were either boiled at 95°C for 5 min, or not boiled, followed by detection of the expression by SDS-PAGE and Coomassie Blue staining (B), and Western blot (C) by using a HA1-specific mAb. The protein molecular weight marker (kDa) (Invitrogen) is indicated on the left.

Since the molecular weight shown in reducing SDS-PAGE would not represent the actual size of the tested proteins, we next sought to detect the conformation of these proteins using non-reducing N-PAGE by removing the reducing agents in both sample and running buffers. As indicated in Fig. 5A, clear bands with high molecular weight were detected in HA-13–263-Fdc, HA-13–263-Fc and HA-13–263-Fd-His proteins, with HA-13–263-Fdc showing the highest molecular weight oligomer, while no clear band was shown in HA-13–263-His protein. Similarly, these bands were detected by a HA1-specific mAb in Western blot (Fig. 5B), indicating their high specificity to the HA1 protein. Comparison of the molecular weight from samples with and without cross-linker showed that the molecular weights of the cross-linker samples for HA-13–263 with Fd and/or Fc were about 1-, 2- or 3-fold higher than that of the corresponding without-cross-linker samples, but the molecular weight of the cross-linker HA-13–263-His was almost the same as that of the without-cross-linker HA-13–263-His (Fig. 5C). These results suggest that the identified neutralizing HA-13–263 fragment fused with Fd and/or Fc tags was able to form conformational structures of dimer, trimer, or oligomer.

**Figure 5:** Detection of conformation of HA-13–263 proteins by native PAGE (N-PAGE) and cross-linker analysis. (A) N-PAGE analysis of expressed HA-13–263 proteins, followed by Coomassie Blue staining and Western blot (B), by using a HA1-specific mAb. The native protein molecular weight marker (kDa) (Invitrogen) is indicated on the left. (C) Cross-linker analysis followed by SDS-PAGE and Coomassie Blue staining of expressed HA-13–263 proteins (with cross-linker). The proteins without cross-linking (w/o cross-linker) were used as the controls. The protein molecular weight marker (kDa) (Invitrogen) is indicated on the left.

### Fragment Containing Residues 13–263 of HA1 with Optimal Conformation Induced a High Level of Cross-neutralizing Antibody Responses

To evaluate the ability of conformational proteins in improving immune responses, we immunized mice using purified HA-13–263 proteins with or without Fd and/or Fc, and compared the IgG antibody response, subtypes and neutralizing antibodies in the collected mouse sera. The results, as shown in Fig. 6A and B, demonstrated that HA-13–263-Fdc and HA-13–263-Fc induced higher titers of IgG antibodies against the HA protein than HA-13–263-Fd-His or HA-13–263-His. While HA-13–263-Fdc induced the highest titer of IgG antibodies, HA-13–263-His induced the lowest antibody responses against the HA protein. Detection of the IgG subtypes indicated that HA-13–263-Fdc and HA-13–263-Fc proteins induced similar higher levels of IgG1 and IgG2a than HA-13–263-Fd-His, while HA-13–263-His elicited the lowest level of IgG1 and IgG2a in the vaccinated mice (Fig. 6C and D). However, PBS control only induced background level of IgG antibody responses and subtypes (Fig. 6).

**Figure 6:** Detection of IgG antibody responses and subtypes by ELISA in HA-13–263 protein-vaccinated mouse sera. PBS was used as the negative control. Ability of IgG binding to HA1 (HA-13–263-His) protein (A) and full-length HA protein (B) was detected using mouse sera from 10 days post-last vaccination. The data are presented as mean A450± SD of five mice per group at various dilution points. Ability of IgG1 (C) and IgG2a (D) antibodies to bind to HA-13–263-His protein was detected using sera from 10 days post-last vaccination. The data are presented as mean A450± SD of five mice per group at various dilution points.

Further evaluation of the neutralizing activity of these proteins in vaccinated mouse sera revealed that all HA-13–263 proteins with Fd and/or Fc were able to induce a significantly higher level of neutralizing antibodies than HA-13–263-His against homologous (AH-HA) and heterologous (HK-HA and 1194-HA) H5N1 pseudoviruses. Specifically, HA-13–263-Fdc and HA-13–263-His induced the highest and lowest neutralizing antibody responses, respectively, against all three H5N1 strains, while HA-13–263-Fc elicited a significantly higher level of neutralizing antibodies than HA-13–263-Fd-His. However, PBS control did not induce neutralizing antibodies against any tested pseudoviruses (Fig. 7A).

**Figure 7:** Comparison of neutralizing antibodies in sera of mice vaccinated with HA-13–263 proteins. Sera were collected at 10 days post-last vaccination. PBS was used as the negative control. (A) Neutralizing antibody titers against HA of homologous AH-HA strain (clade 2.3.4) and heterologous A/Hong Kong/156/97 (HK-HA, clade 0) and A/VietNam/1194/2004 (1194-HA, clade 1) strains of H5N1 pseudovirus. The data are presented as mean NT_50_± SD from five mice per group. * indicates significant difference (*P*<0.05), respectively, between HA-13–263-Fdc, HA-13–263-Fc, or HA-13–263-Fd-His vaccination groups and HA-13–263-His group or PBS control for the three H5N1 pseudoviruses. (B) Neutralizing antibody titers against heterologous strains of A/VietNam/1194/2004 (VN/1194, clade 1) and A/Shenzhen/406H/06 (SZ/406H, clade 2.3.4) H5N1 live viruses. The titers of neutralizing antibodies are presented as mean ± SD of five mice per group. * indicates significant difference (*P*<0.05), respectively, between HA-13–263-Fdc, HA-13–263-Fc, or HA-13–263-Fd-His vaccination groups and HA-13–263-His group or PBS control for both VN/1194 and SZ/406H viruses. The dotted line shows the limit of detection.

Neutralizing activities induced by these proteins were further evaluated by a live-virus- based neutralization assay. Similarly, HA-13–263-Fdc and HA-13–263-His elicited the highest and lowest neutralizing antibody responses, respectively, against two (VN/1194 and SZ/406H) H5N1 live viruses tested, while HA-13–263-Fc and HA-13–263-Fd-His induced similarly high level of neutralizing antibodies. The PBS control group only induced a background level of neutralizing antibodies against tested H5N1 viruses (Fig. 7B). These results suggest that HA-13–263 proteins with appropriate polymeric conformational structures were capable of inducing a significantly higher level of antibody responses and cross-neutralizing activity than monomeric protein covering the same neutralizing fragment against H5N1 virus infections.

### Fragment Containing Residues 13–263 of HA1 Proteins with Optimal Conformation Significantly Increased Mouse Survival Rate and Decreased Body Weight Loss after Challenge with Variant H5N1 Viruses

To demonstrate the ability of HA-13–263 proteins with suitable polymeric conformation to promote greater cross-protection than protein monomer, mice vaccinated with the above fusion proteins were challenged with VN/1194 (clade 1) and SZ/406H (clade 2.3.4) H5N1 viruses 10 days post-last vaccination and observed daily for two weeks for survival and body weight change. As shown in Fig. 8A and B, HA-13–263-Fdc protein completely cross-protected all vaccinated mice against VN/1194 and SZ/406H virus challenge. HA-13–263-Fc and HA-13–263-Fd-His protected all vaccinated mice against challenge of SZ/406H strain, and both proteins could protect 80% of the vaccinated mice against VN/1194 virus challenge. Compared with the HA-13–263 proteins fused with Fd and/or Fc, the protein HA-13–263-His provided much lower protection rate. No mice in the PBS control group survived the challenge of two virus strains after day 10.

**Figure 8:** Comparison of cross-protective activity of HA-13–263 proteins against lethal H5N1 virus challenge. PBS was used as the control. Survival rate (%) of mice vaccinated with HA-13–263 proteins challenged with lethal dose of H5N1 virus from VN/1194 (clade 1) (A) and SZ/406H (clade 2.3.4) (B). * indicates significant difference (*P*<0.05), respectively, between HA-13–263-Fdc and HA-13–263-His group, or PBS control, for VN/1194 virus, and between HA-13–263-Fdc, HA-13–263-Fc, or HA-13–263-Fd-His vaccination groups and HA-13–263-His group, or PBS control for SZ/406H virus. Percentage of body weight change (%) of HA-13–263-vaccianted mice after challenge with VN/1194 (C) and SZ/406H (D) H5N1 virus was shown.

Only slight body weight loss (less than 3%) was found on day 6–8 in the mice vaccinated with HA-13–263-Fdc after challenge with VN/1194 and SZ/406H viruses. Mice vaccinated with HA-13–263-Fc and HA-13–263-Fd-His proteins after challenge with SZ/406H were able to regain normal body weight. In addition, mice from the HA-13–263-Fc and HA-13–263-Fd-His vaccination groups showed a slightly higher level of body weight loss (around 6% on day 8 post-challenge) than those from HA-13–263-Fdc vaccination group after challenge with VN/1194 virus. In contrast, mice vaccinated with HA-13–263-His demonstrated a significant loss of body weight, particularly during day 6–12, after respectively challenge with VN/1194 and SZ/406H virus strains. However, all mice from the PBS control group indicated an obvious and continual decrease of body weight after day 2, all of which reaching >25% severe weight loss by day 8–10 post-challenge (Fig. 8C and D). The mice that lost greater than 25% of their initial body weight were humanely euthanized.

The above results suggested that HA-13–263 proteins with suitable polymeric conformation, particularly the one fused with Fd and Fc, could significantly protect vaccinated mice against various H5N1 virus challenges.

### Fragment Containing Residues 13–263 of HA1 Proteins with Optimal Conformation Significantly Reduced Virus Titers in the Mice Infected with Divergent Strains of H5N1 Virus

The cross-protective effect induced by HA-13–263 proteins fused with or without Fd and/or Fc was further evaluated by detection of viral titers in the lung tissues of vaccinated mice challenged with H5N1 virus. As shown in Fig. 9, a significantly lower level of virus titers was detected in the mice vaccinated with HA-13–263-Fdc, HA-13–263-Fc and HA-13–263-Fd-His proteins than those vaccinated with HA-13–263-His protein after challenge with both VN/1194 and SZ/406H viruses (*P*<0.05). However, virus titer in the PBS control group was still significantly higher than that of the HA-13–263-His vaccination group. These results suggested that the HA-13–263 proteins with suitable polymeric conformation after the addition of Fd and/or Fc can induce strong cross-protection against divergent H5N1 virus challenge.

**Figure 9:** Comparison of viral titers in virus-challenged lung tissues of mice vaccinated with HA-13–263 proteins. Viral titers of VN/1194 (clade 1) and SZ/406H (clade 2.3.4) H5N1 viruses were determined in the lung tissues of the mice vaccinated with HA-13–263 proteins, respectively, collected on 5 day post-challenge. Mice injected with PBS were used as the negative control. * indicates significant difference (*P*<0.05), respectively, between HA-13–263-Fdc, HA-13–263-Fc, or HA-13–263-Fd-His vaccination groups and HA-13–263-His or PBS control group. The data are expressed as mean ± SD of viral titers 50% tissue culture infective dose (Log_10_TCID_50_/g) of lung tissues from five mice per group. The limit of detection is 1.5 Log_10_TCID_50_/g of tissues.

## Discussion

The HAPI H5N1 virus has continuously crossed the species barrier and frequently infected humans since the confirmed human case reported to WHO in 2003 (http://www.who.int/influenza/human_animal_interface/EN_GIP_20120810CumulativeNumberH5N1cases.pdf). Although the ability to generate highly transmissible forms of H5N1 in the laboratory enables investigators to further elucidate the mechanism of virus transmission, such advancement poses a considerable threat to public health, raising concerns over issues of biosafety and dual-use research [22]–[26]. Thus, the search for readily available effective vaccines is more than justified to prevent seasonal epidemics and prepare for unpredicted H5N1 virus infections [27].

Currently, a variety of vaccines have been developed specifically targeting H5N1 virus in the form of inactivated virus-, live virus-, DNA-, and viral vector-based vaccines, some of which have shown efficacy against virus infection in preclinical or clinical trials [3], [28]–[30]. Reports have demonstrated that vaccination with drifted variants of avian H5 HA protein elicits a broadened antibody response that is protective against challenge with homologous or drifted live H5 influenza virus [31]. A consensus-HA-based DNA vaccine is also seen to protect mice against divergent H5N1 influenza viruses [32]. In addition, a live attenuated modified vaccinia Ankara (MVA) vector vaccine expressing influenza H5N1 HA induces substantial cross-clade protective immunity in vaccinated animals [33]. A Vero cell-derived, whole virus clade 2 H5N1 influenza vaccine is now in phase I/II study for safety and immunogenicity testing in healthy adults in Hong Kong and Singapore, and shows high tolerance and immunogenicity after two vaccinations with induction of a cross-neutralizing antibody response [34]. Nevertheless, because of the continual and frequent mutation of H5N1 virus, particularly the viral HA protein, currently available H5N1 vaccines are facing significant efficacy challenges against new virus strains, making it extremely important to identify critical neutralizing regions for utilization as targets to develop effective and safe vaccines against ever-changing divergent virus strains.

As a receptor binding and fusion protein, the HA of influenza virus plays an important role in initiating viral infection. The receptor-binding domain of H5N1 HA determines the species of sialic acid receptors in α(2,3) linkages [9], [12]. HA, particularly its HA1 subunit, is the main region for the induction of neutralizing activity against influenza virus infection [15], [33], [35] and can be used for development of subunit influenza vaccine. Indeed, we previously demonstrated that a recombinant protein containing the full-length HA1 of H5N1 could elicit neutralizing antibody responses in the immunized mice [15], confirming that the HA1 subunit contains important neutralizing epitopes. However, recent study on the development of SARS vaccine has raised a serious concern about the safety of using the full-length S protein of SARS-CoV as a vaccine since the non-neutralizing regions in the S protein could induce harmful immune responses in the vaccinated animals [36]. Therefore, it is essential to identify the CND for designing an effective influenza vaccine containing the major neutralizing domain in HA1. We therefore constructed six truncated recombinant fragments covering partial or full-length RBD or other regions in HA1 (Fig. 1) for immunization of mice. Although all six truncated protein fragments were able to induce strong HA1-specific antibodies in the vaccinated mice, only the one containing residues 13–263 covering full-length RBD induced a significantly higher level of neutralizing antibodies against pseudotyped H5N1 virus than other fragments (Fig. 3), suggesting that this fragment contains the CND in HA1. Comparison of the amino acid sequences of the identified CND revealed high similarity among hundreds of H5N1 strains causing human and avian diseases (data not shown), suggesting that the identified CND has a high potential to be developed as a universal candidate vaccine particularly against H5N1.

Native influenza HA protein is polymerized as trimer [9]. It seems that recombinant HA fragments themselves cannot easily form functional, conformational trimeric or oligomeric structures, while the formation of these functional molecules of HA may be introduced through the addition of extraneous sequences [14], [37]. A trimeric HA could be formed by fusing HA with a trimeric GCN4pII heptad repeat sequence derived from wild-type dimeric GCN4 repeat found in *Saccharomyces cerevisiae* [14]. The Fd sequence, the C-terminal domain of T4 fibritin, is often applied as an artificial trimerization domain, and is thus required to form fibritin trimer structure [38]. Recombinant proteins conjugated with this motif have been shown to form stable trimers with improved antiviral activity [39]. Fc is utilized as another motif to promote oligomeric conformation of expressed proteins for the purpose of increasing immunogenicity of recombinant proteins [37]. Therefore, we further constructed three additional recombinant proteins based on the identified neutralizing region fused with Fd and Fc by fusing the HA fragment with Fd-His, Fc or His, respectively, and the conformation of these proteins was subsequently evaluated. As expected, HA-13–263 protein with Fd and Fc (HA-13–263-Fdc) was able to form an oligomeric structure with the highest molecular weight, while those fused with Fc (HA-13–263-Fc) or Fd-His (HA-13–263-Fd-His) formed different polymeric conformations, including dimer or trimer, with relatively lower molecular weight. However, the protein without fusion with Fd or Fc (HA-13–263-His) did not form polymeric conformational structure, but remaining the monomeric form (Fig. 4 and 5). Thus, our results further emphasize the importance of adding foreign motif in promoting oligomerization of HA.

It is believed that proteins capable of maintaining native trimeric or oligomeric structure of HA would likely induce stronger immune responses than monomers [14], [37], [40]. To determine conformational structure covering the identified critical neutralizing region of HA1 in enhancing immune responses and cross-protective immunity, we first immunized mice using these fusion proteins and then compared antibody response and neutralizing antibodies in addition to the evaluation of cross-protection against two different strains of H5N1 virus in cell cultures *in vitro* and in mouse models *in vivo*. It was found that HA-13–263-Fdc protein with the highest molecular weight oligomer induced the strongest neutralizing antibody responses and cross-protection against challenges by two tested H5N1 strains including clade 1 and clade 2.3.4, followed by lower molecular weight polymers HA-13–263-Fc (mainly dimer) and HA-13–263-Fd (mainly trimer). The monomeric HA-13–263-His protein induced much lower level of neutralizing antibody response and protection than the HA-13–263 proteins fused with Fd and/or Fc (Fig. 6–9). The above data indicate that while the trimeric HA-13–263-Fd-His protein may elicit stronger protection than the HA-13–263-His monomer, the oligomeric HA-13–263 with Fd and Fc promoted this protection. The Fc fragment in an immunogen can enhance its immunogenicity, possibly by prolonging half-life of the immunogen, or interacting with Fc receptor (FcR) on antigen presenting cells (APCs) [41]-[43]. The immunogen with both Fd and Fc can form an oligomer with higher molecular weight than the dimer formed by HA-13–263-Fc. Therefore, HA-13–263-Fdc may have even longer half-life than HA-13–263-Fc, thus demonstrating stronger effect on induction of immune responses. It is noted that neither Fc alone nor Fd alone is able to induce HA-specific antibody responses, and that none of the expressed HA proteins induced antibody responses against HAs of seasonal influenza A viruses including H1N1 and H3N2 (data not shown), further confirming the high specificity of our recombinant proteins to the HA of H5N1. Our results further demonstrated that influenza H5N1 HA-specific proteins with polymeric conformational structures may significantly enhance cross-protective immunity against divergent strains of H5N1 influenza virus infections [14], [40], [44].

In summary, we identified a CND, which contains the RBD, in the HA1 of H5N1 virus. Addition of Fd and Fc to this CND resulted in the formation of oligomeric conformation, which could induce highly potent neutralizing antibody responses and cross-protection against two tested H5N1 strains covering clade 1 and clade 2.3.4, respectively. These results suggest that the identified CND of H5N1 HA1 in an optimal conformation has a great potential to be further developed as an effective and safe influenza vaccine for preventing H5N1 infection and similar strategy can be used for designing vaccines against other emerging or re-emerging viral pathogens with class I glycoproteins.

## Materials and Methods

### Ethics Statement

The animal studies were carried out in strict accordance with the recommendations in the Guide for the Care and Use of Laboratory Animals of the National Institutes of Health and State Key Laboratory of Pathogen and Biosecurity, Beijing Institute of Microbiology and Epidemiology. The protocol was approved by the Committee on the Ethics of Animal Experiments of the New York Blood Center (Permit Number: 322). All experiments related to the influenza viruses were performed in approved biosafety level 3 (BSL-3) laboratories or BSL-3 animal facilities of Beijing Institute of Microbiology and Epidemiology of China (Permit Number: PBS012).

### Construction, Expression and Purification of Recombinant HA1 Proteins

The construction, expression and purification of recombinant HA proteins were done as previously described [15]. Briefly, genes encoding truncated HA1 of A/Anhui/1/2005(H5N1) (AH/1, accession No. ABD28180) with Fd were amplified by PCR using a recombinant HA1 plasmid fused with Fd and Fc (HA1-Fdc) as the template. A 6× Histidine (His) tag was added at the C-termini of HA-13–263 (HA-13–263-His) and HA-13–263-Fd (HA-13–263-Fd-His), respectively, for easy purification of the proteins. Amplified gene fragments were digested by EcoR I and Bgl II restriction enzymes and inserted into the pFUSE-hIgG1-Fc2 expression vector (hereinafter named Fc, InvivoGen, San Diego, CA). The plasmid encoding residues 13–263 of HA1 with Fc (HA-13–263-Fc) was constructed by inserting digested HA-13–263 fragment directly into the Fc vector. Recombinant plasmids were then transfected into 293T cells (ATCC, Manassas, VA) seeded 24 h before transfection. Culture medium was replaced by serum-free DMEM (Invitrogen, Carlsbad, CA) 10 h later, and supernatant containing expressed proteins was collected 72 h post-transfection. The recombinant proteins were purified by Protein A affinity chromatography (GE Healthcare, Piscataway, NJ) (for proteins with Fc) or Ni-NTA Superflow (Qiagen, Valencia, CA) (for proteins with His tag), according to the manufacturers’ instructions. Constructed recombinant fragments were illustrated in Fig. 1 and 4A.

### Characterization of Recombinant Proteins by SDS-PAGE, N-PAGE, Cross-linker and Western Blot Analysis

The purified proteins were first analyzed by SDS-PAGE and Western blot as previously described [15], [45]. Briefly, the proteins were either non-boiled or boiled at 95°C for 5 min and separated by 10–20% Tricine gels (Invitrogen), which were then stained with Coomassie Blue or transferred to nitrocellulose membranes for Western blot analysis. After blocking with 5% non-fat milk in PBST overnight at 4°C, the blots were incubated with a HA1-specific mAb (1∶500) developed in our laboratory for 1 h at room temperature. After three washes, the blots were then incubated with horseradish peroxidase (HRP)-conjugated goat anti-mouse IgG (1∶5,000, Invitrogen) for 1 h at room temperature. Signals were visualized with ECL Western blot substrate reagents and Amersham Hyperfilm (GE Healthcare).

For N-PAGE analysis, the proteins were first separated by 6% N-PAGE gels using N-PAGE sample buffer and running buffer (Invitrogen), followed by the same protocols as above. For protein cross-linker detection, 4.5 µg of a purified protein was mixed with 20 µl of 0.1% glutaraldehyde (final concentration 4 mM) and left at room temperature in the dark for 2 h before SDS-PAGE and Coomassie Blue staining as described above.

### Mouse Vaccination and Sample Collection for Antibody and Neutralization Detection

Four- to six-week-old female BALB/c mice were prime-vaccinated subcutaneously (s.c.) with 20 µg/mouse of a recombinant HA protein fragment formulated with Montanide ISA 51 adjuvant (SEPPIC, Fairfield, NJ) and boosted twice with 10 µg/mouse of immunogen with adjuvant at 3-week intervals. Control mice were s.c. injected with the same volume of PBS with adjuvant. Sera were collected at 10 days post-last vaccination to detect HA-specific IgG antibodies, subtypes and neutralizing antibodies.

### ELISA

Collected mouse sera were analyzed for HA-specific antibody responses by ELISA as described previously [15]. Briefly, 96-well ELISA plates were respectively precoated with truncated HA1 protein fragments or full-length HA protein (eEnzyme, Gaithersburg, MD) overnight at 4°C and blocked with 2% non-fat milk for 2 h at 37°C. Serially diluted mouse sera were added to the plates and incubated at 37°C for 1 h, followed by four washes. Bound antibodies were incubated with HRP-conjugated goat anti-mouse IgG (1∶2,000, Invitrogen), anti-mouse IgG1 (1∶2,000, Bethyl Laboratories, Montgomery, TX) or anti-mouse IgG2a (1∶2,000, Invitrogen) for 1 h at 37°C. The reaction was visualized by substrate 3,3′,5,5′-tetramethylbenzidine (TMB) (Invitrogen) and stopped by 1N H_2_SO_4_. The absorbance at 450 nm (A450) was measured by ELISA plate reader (Tecan, San Jose, CA).

### Pseudovirus Neutralization Assay

Neutralizing activity in collected mouse sera was performed using our established pseudovirus neutralization assay as previously described [46]. Briefly, 293T cells were co-transfected with a plasmid encoding Env-defective, luciferase-expressing HIV-1 genome (pNL4-3.luc.RE) and each of the plasmids encoding HA of homologous AH-HA (clade 2.3.4) and heterologous H5N1 containing HK-HA (clade 0) and 1194-HA (clade 1). Exogenous bacterial neuraminidase (NA) (Sigma, St. Louis, MO) was added 24 and 48 h later, and supernatant was harvested 72 h post-transfection for single-cycle infection. Pseudovirus-containing supernatant was incubated with serially diluted mouse sera at 37°C for 1 h before adding to 293T cells. Fresh medium was added 24 h later, and the culture was continued for 72 h. Cells were lysed by cell lysis buffer (Promega, Madison, WI) and transferred to 96-well luminometer plates. Luciferase substrate (Promega) was added, and relative luciferase activity was determined by Ultra 384 luminometer (Tecan). The neutralization of HA pseudovirus was calculated [47] and presented as NT_50_.

### Live Virus-based Neutralization Assay

Neutralizing antibody titers of mouse sera were further detected by a live virus-based neutralization assay, as previously described, with some modifications [15]. Briefly, serial diluted mouse sera were incubated with 100 TCID_50_ of H5N1 influenza virus containing VN/1194 (clade 1) or SZ/406H (clade 2.3.4) for 2 h at 37°C prior to addition to monolayers of Madin-Darby canine kidney (MDCK) cells. Virus supernatant was removed and replaced with fresh medium. The virus-infected cells were incubated for 72 h at 37°C. Infectivity was identified by the presence of cytopathic effect (CPE) on day 4, and the titer was calculated by the Reed-Muench method.

### Virus Challenge

Five groups of female BALB/c mice at 6–8-weeks were respectively s.c. vaccinated with 20 µg/mouse of recombinant proteins containing HA-13–263 of AH/1 fused with Fc (HA-13–263-Fc), Fd (HA-13–263-Fd), Fd plus Fc (HA-13–263-Fdc) or without Fd and Fc (HA-13–263-His), plus adjuvant, and boosted twice at 3-week intervals. Vaccinated mice were intranasally (i.n.) infected with 50% lethal dose (5 LD_50_) of VN/1194 (clade 1) or SZ/406H (clade 2.3.4) H5N1 virus, respectively, at 10 days post-last vaccination. Infected mice were observed daily for 14 days for the clinical signs, including body weight loss, and survival rate was accordingly calculated. Mice that lost greater than 25% of body weight were euthanized. Five mice per group were sacrificed on day 5 post-challenge, and lung samples were collected for virological analysis. All of the vaccination, infection, and euthanasia procedures were performed under anesthesia with isoflurane, and lung tissue harvest was performed only after the mice have been euthanized.

### Virus Titer Detection

Virus titers were detected as previously described [15], [48]. Briefly, lung tissues from euthanized mice were aseptically removed and homogenized in minimal essential medium (MEM) plus antibiotics to achieve 10% (w/v) suspensions of lungs. In 96-well cell culture plates, ten-fold serial dilutions of samples were added to monolayers of MDCK cells in quadruplicate and allowed to absorb for 2 h at 37°C in the presence of 5% CO_2_. Supernatants were then removed and replaced with MEM plus antibiotics, and MDCK cells were incubated as above for 72 h. Viral CPE was observed daily, and virus titer was determined by HA test. For the HA test, 50 µl of 0.5% turkey red blood cells (Lampire Biological Laboratories, Pipersville, PA) were added to 50 µl of cell culture supernatant and incubated at room temperature for 30 min. Wells containing HA were scored as positive. The virus titer was calculated by the Reed and Muench method and expressed as Log_10_TCID_50_/g of lung tissues.

### Statistical Analysis

Values were presented as mean with SD. Statistical significance among different groups was calculated by Student’s *t* test using *Stata* statistical software. *P* values less than 0.05 were considered significant.
